# Role of homocysteine in the development of cardiovascular disease

**DOI:** 10.1186/1475-2891-14-6

**Published:** 2015-01-10

**Authors:** Paul Ganguly, Sreyoshi Fatima Alam

**Affiliations:** College of Medicine, Alfaisal University, Riyadh, Kingdom of Saudi Arabia; King Faisal Specialized Hospital and Research Centre, Riyadh, Kingdom of Saudi Arabia

## Abstract

It is well known that neuronal damage following a stroke has been attributed to the over stimulation of excitatory amino acids such as glutamate and aspartate through activation of NMDA receptors. The brain is exposed to most of the constituents of plasma including homocysteine as a result of the disruption of the blood–brain barrier after stroke, head trauma and stress. The question, therefore, arises as to whether or not homocysteine is able to selectively stimulate the release of excitatory amino acids in stroke. This review article will address the importance of homocysteine in nervous system specifically how these amino acids may trigger the release of catecholamines. Our data will thus strengthen the view that a mechanism for the association of hyperhomocysteinemia with increased brain lesion in stroke. As hypothalamus also controls the cardiac function via sympathetic system, the contractility of heart will be compromised. Homocysteine is also known to mediate cardiovascular problems by its adverse effects on cardiovascular endothelium and smooth muscle cells with resultant alterations in subclinical arterial structure and function. The present review will thus summarize both central and peripheral effects of homocysteine and will highlight some of the controversies associated with hyperhomocysteinemia-induced cardiovascular problems.

## Introduction

Homocysteine has been under a lot of speculation since its discovery in 1932. Its chemical properties showed a similarity to cysteine, hence the name homocysteine. The heating of the amino acid methionine with sulphuric acid led to this amino acid of interest. The importance of this discovery cannot be emphasized on without alluding to the 1955 Nobel Prize in Chemistry, awarded to Vincent du Vigneaud “For his work on biochemically important sulphur compounds, especially for the first synthesis of a polypeptide hormone” [1]. Recent years have shown a dramatic increase in research towards the better understanding of the notoriety of this amino acid of interest (Figure 1).

**Figure 1:** **Structure of homocysteine.**

Homocysteine, a sulfhydryl-containing amino acid, is an intermediate product in the normal biosynthesis of the amino acids methionine and cysteine [2]. It is an amino acid produced via demethylation of dietary methionine, which is abundant in animal protein [3]. It is present in plasma in four different forms: around 1% circulates as free thiol, 70–80% remains disulphide-bound to plasma proteins, mainly albumin and 20–30% combines with itself to form the dimer homocysteine or with other thiols [4]. Homocysteine is a key determinant of the methylation cycle [5]. It is methylated to methionine, which undergoes S-adenosylation and forms S-adenosylmethionine (SAM) [5]. S- adenosylmethionine is the principal methyl donor for all methylation reactions in cells [5]. Condensation of methionine with ATP, leads to the formation of SAM (S- Adenosylmethionine) [6]. The methyl group attached to the tertiary sulphur of SAM can be transferred and therefore can cause methylation of other substances. This methylation is accompanied by energy loss, so this reaction is irreversible. The demethyation reaction leads to the formation of SAH (S- adenosylhomocysteine) [6]. SAH is a thioether (a sulfur bonded to two alkyl or aryl groups) analogous to methionine. The SAM-to-SAH ratio defines the methylation potential of a cell [5]. Hydrolysis of SAH leads to the formation of homocysteine and adenosine [6]. This homocysteine can be used in one of two ways:

- In case of methionine deficiency, homocysteine can be re-methylated to form methionine [6]. The enzyme N5, N10-methylenetetrahydrofolate reductase converts homocysteine to methionine [2].
- In presence of sufficient methionine, homocysteine is instead used to produce cysteine [6]. Cystathionine-β-synthase is an enzyme (with pyridoxine (vitamin B_6_) as an essential cofactor) that converts homocysteine to cysteine [2]. Homocysteine is synthesized from the essential amino acid methionine, therefore cysteine is not an essential amino acid as long as sufficient methionine is available [6].

### Biochemical basis of hyperhomocysteinemia

While the present analysis will provide an insight into cause-and-effect of hyperhomocysteinemia and cardiovascular diseases, the potential role of nutritional homocysteine are great and the readers are referred to other articles dealing with nutritional therapies for managing homocysteine.

The definition of hyperhomocysteinemia differs between studies [2]. Hyperhomocysteinemia is defined as a medical condition characterized by an abnormally high level (above 15 μmol/L) of homocysteine in the blood [7]. Total concentration of homocysteine in plasma of healthy humans (fasting) is low and its level is between 5.0 and 15.0 μmol/L when assessed with the use of HPLC, or 5.0-12.0 μmol/l when immunoassay methods are used [8]. When the level is between 16-30 μmol/L it is classified as moderate, 31-100 μmol/L is considered intermediate and a value above 100 μmol/L is classified as severe hyperhomocysteinemia [4]. There are two types of hyperhomocysteinemia: (1) the rare but severe forms are due to major genetic mutations of the enzymes implicated in homocysteine metabolism; (2) the more common forms cause moderately elevated homocysteine levels related to a pathogenesis such as genetic and environmental factors [2].

Hyperhomocysteinemia may arise from genetic defects of enzymes involved in homocysteine metabolism. The enzymes involved can be 5, 10-methylene tetrahydrofolate reductase, methionine synthase, and cystathionine-β-synthase [9]. The most common one that is detected worldwide and has a high incidence in different populations, is single nucleotide polymorphisms of 5,10-methylene tetrahydrofolate reductase which has been associated with mild (13–24 μM) and moderate (25–60 μM) hyperhomocysteinemia [9]. Hankey et al. [4] stated that the most common enzyme defect associated with moderately raised total homocysteine is a point mutation (C-to-T substitution at nucleotide 677) in the coding region of the gene for MTHFR, which is associated with a thermo labile MTHFR variant that has about half-normal activity [4]. The most common of the genetic causes of severe hyperhomocysteinemia and classic homocystinuria (congenital homocystinuria) is believed to be homozygous deficiency of CβS (cystathionine-β-synthase) which results in an increase of up to 40-fold in fasting total homocysteine. Other rarer causes of severe hyperhomocysteinemia are considered to be homozygous deficiency of MTHFR, deficiency of methionine synthase, and impaired activity of methionine synthase due to genetic disorders of vitamin B_12_ metabolism [4].

Hyperhomocysteinemia can also arise from nutritional deficiencies of folate, vitamin B_6_, and vitamin B_12_ [9]. Blood levels of folate, vitamin B_12_ and to a lesser extent, vitamin B_6_ are related inversely to total homocysteine; therefore a person with a nutritional deficiency that leads to low blood concentrations of the aforementioned is at increased risk of hyperhomocysteinemia [4, 9]. Several diseases such as renal and thyroid dysfunction, cancer, psoriasis, and diabetes as well as various drugs, alcohol, tobacco, coffee, older age and menopause, are believed to be associated with moderately elevated homocysteine concentrations [2]. A rise in serum creatinine also leads to a rise in fasting total homocysteine [4]. The major route of homocysteine clearance from plasma is the kidney, and the rise is due to defective metabolism of homocysteine by the kidney [4]. Total homocysteine levels are found to be considerably higher in patients with chronic renal disease than the moderately raised concentrations commonly found in patients with atherothrombotic vascular disease, and this may be the probable cause that contributes to the high incidence of vascular complications in patients with chronic renal failure [4]. Plasma homocysteine concentrations can be increased by various drugs and diseases that interfere with folate, vitamin B_6_, and B_12_ metabolism, hence an abnormal homocysteine concentration may have a probable use as a diagnostic aid for some of these conditions [4].

There has been an indication towards a significant correlation between hyperhomocysteinemia and cardiovascular disease and its complications such as heart attacks and strokes [8]. It is believed that hyperhomocysteinemia leads to endothelial cell damage, reduction in the flexibility of vessels, and alters the process of haemostasis [8]. Hyperhomocysteinemia may lead to an enhancement of the adverse effects of risk factors like hypertension, smoking, lipid and lipoprotein metabolism, as well as promotion of the development of inflammation [8]. The prevalence of hyperhomocysteinemia may vary significantly between populations, and most likely depend on age, diet, and genetic background as well [2]. Increasing age, male sex, smoking, coffee consumption, high blood pressure, unfavourable lipid profile, high creatinine and faulty diet are some of the factors associated with increased homocysteine levels [10]. On the other hand, physical activity, moderate alcohol consumption, good folate and vitamin B_12_ status are associated with lower homocysteine levels. Vegetarians may be at a higher risk of hyperhomocysteinemia due to low plasma B_12_ levels but the difference is likely to be insignificant [10].

The SAM-to-SAH ratio defines the methylation potential of a cell as mentioned before. Hyperhomocysteinemic states tend to decrease this ratio, leading to decreased methylation potential [5]. There is some evidence that indicates that homocysteine can lead to global DNA hypomethylation. It may also suppress transcription of cyclin A in endothelial cells [5]. This is a gene-specific effect. In the core promoter, it causes demethylation of a CpG site and this eliminates the binding of methyl CpG-binding protein 2. This in turn, limits HDAC (Histone deacetylases) binding. Therefore this causes acetylated H3 and H4 histones to accumulate and to suppress gene expression [5]. DNA hypomethylation and histone acetylation are associated with transcriptional permissive chromatin [5]. The open conformation of chromatin may allow increased access by repressor proteins, leading to transcriptional suppression. To account for changes in apoA-1 and apoA-IV in hyperhomocysteinemia, similar epigenetic regulatory mechanisms have been reported [5]. On the contrary, homocysteine-induced DNA hypomethylation of their promoters causes some genes to be up regulated, for example, the homocysteine induction increases p66shc expression in endothelial cells, and this correlates with promoter hypomethylation thus contributing to oxidant stress [5].

### The homocysteine and the nervous system

In the last decade, epidemiological observations have pointed towards a plausible association between hyperhomocysteinemia and CNS neurodegenerative disorders. Several studies demonstrated that homocysteine is capable of triggering neuronal damage via oxidative stress, DNA damage and activation of pro-apoptotic factors in cell cultures or animal models [9]. In an experiment, SH-SY5Y neuroblastoma cells were modified to act as neuronal cells, by incubating them with retinoic acid, which induced their differentiation towards a neuronal-like phenotype [9]. This was followed by incubation with/without D,L-homocysteine in a concentration range from 20 μM to 80 μM [9]. The exposure to homocysteine induced a time and concentration dependent reduction of cell viability in comparison with controls. The highest cytotoxicity was portrayed by 80 μM homocysteine which produced 80% of cell death after 5 days of incubation [9]. A significant reduction of cell viability to 35% was also observed after 5 days of incubation with 40 μM homocysteine. Cell exposure to homocysteine for a period of 3 days did not induce any significant change in Reactive Oxygen Species (ROS) levels, but incubation with homocysteine for 5 days resulted in a 4.4-fold increase in ROS production [9]. Homocysteine notably triggered significant levels of genotoxic stress which was indicated by the assessment of DNA fragmentation by Comet assay. But the levels of genotoxic stress was significant only after a longer time of exposure, as shown by the number of Comet positive cells, which was significantly increased only after 5 days of incubation with homocysteine [9]. Bax and Bcl-2 mRNA levels in cells showed an increase by two-fold and 14-fold, respectively, in the case of 5 days exposure to homocysteine [9]. A time-dependent effect of homocysteine was also evident. The mRNA levels for the cyclins D1, E1, and A1 were increased by two-fold, six-fold, and five-fold, respectively, in cells exposed to homocysteine for 3 days, but the mRNA levels in case of cyclin B1 were not affected in the 3 day period [9]. The mRNA levels of all cyclins returned to the basal levels after 5 days of incubation with homocysteine. A decrease in both mRNA and protein level, of p21, another key protein regulator of DNA damage induced cell death, was noted after 3 days of incubation with homocysteine, followed by a dramatic p21 up-regulation and protein synthesis at 5 days . Further down the timeline, a significant upregulation of p16 was observed, concomitantly with the reduction by 35% of phosphorylated pRB [9]. These proteins are check-point regulators of G1-S phase progression through the inhibition of cyclin D-cdk4 complex and the direct binding and sequestration of the transcription factor E2F, respectively [9]. Therefore, this indicates the arrest of cell cycle at G1 phase [9]. The results suggest that prolonged exposure to mildly elevated homocysteine concentrations triggers oxidative and genotoxic stress in neuronal-like cells [9].

A) The effect of homocysteine on the brain:

By adulthood, the folate related enzymes involved in purine and pyrimidine synthesis, decline almost tenfold. Hence, this leads us to believe that the provision of methyl groups for SAM and methylation reactions coupled with recycling of homocysteine through methionine synthase may be dominant function of adult brain folate metabolism [11]. The brain has a limited capacity for homocysteine metabolism. Folate plays an important role in the brain so a crucial mechanism is in play to protect the brain from folate deficiency. The level of 5 tetrahydrofolate in the cerebrospinal fluid is 3 times that of the plasma level and there exists an active process to maintain it [11]. Methionine synthase is the only enzyme in the brain (neural tissue) that is capable of converting homocysteine to methionine. Cobalamin is a cofactor (hence essential) [11].

The brain tissue utilizes three mechanisms to maintain a low level of homocysteine [11]:

1. Efficient recycling through cobalamin dependent methionine synthase (given an adequate supply of cobalamine and folate),
2. Catabolism through cystathione beta synthase to cystathione a non-noxious product,
3. Export to external circulation [11].

In the brain and elsewhere disruption of homocysteine metabolism may result from nutritional imbalance, genetic defects or as a result of drug therapy [11].

B) The direct effect of homocysteine on the nervous system:

The action of homocysteine as a neurotransmitter: homocysteine and its related compounds may have a role as an excitatory agonist on the NMDA subtype of glutamate receptors and recent evidence also points to the involvement of NMDA modulatory sites [11]. It has also been shown that homocysteine, besides acting as a partial agonist at glutamate receptors also acts as a partial antagonist of glycine co-agonist site of the NMDA receptor [11]. In the presence of normal glycine levels and normal physiological conditions homocysteine does not cause toxicity below millimolar concentrations. However in case of a head trauma or stroke, there is an elevation in glycine levels in which instance the neurotoxic effect of homocysteine as an agonist outweighs its neuroprotective antagonist effect. This may cause neuronal damage via calcium ion influx or free radical generation [11].

One evaluative experiment to discover the direct effect of homocysteine on the central nervous system involved local application of homocysteine by two different methods of drug delivery to the central nervous system of rats- pressure ejection and ionophoresis [12]. Extracellular recordings were taken from neurons of cerebral cortex, cerebellum and midbrain. The recordings after either method of administration portrayed a dose-dependent increase in neuronal activity by D, L-homocysteine and L-glutamate in 67% of cells tested with both drugs. The similarity in the dose required of D,L-homocysteine and L-Glutamate, points out that D,L-homocysteine seems to be as potent as the latter. This data indicates that homocysteine seems to have an excitatory action on neurons, and this finding may account for neurological symptoms associated with disorders of amino acid metabolism [12]. Some studies also suggest that elevated homocysteine levels may be associated with alterations in mental health such as cognitive impairment, dementia, depression, Alzheimer’s and Parkinson’s disease [2, 11].

### Homocysteine and cardiovascular disease

Cardiovascular diseases (CVD) as the name suggests, comprise of diseases of the heart and blood vessels [13]. Cardiovascular disease is believed to account for one third of all deaths worldwide, and the prevalence is still on the rise [13]. CVD is among the diseases with multiple contributing factors, hence making it difficult to pinpoint a particular factor alone. The main factor that is of relevance to this study is homocysteine. Coronary artery disease is the narrowing or blockage of the arteries and vessels that supply oxygen and nutrients to the heart [10]. The severity of coronary artery disease is classified as single vessel, double vessels and triple vessels disease using the Gensini scoring system [10]. Homocysteine has been recognized as a risk factor as early as 1990s, for the presence of atherosclerotic vascular disease and hypercoagulability states [10]. Subgroup analyses conducted in a study also showed that elevated homocysteine was associated with higher risk of coronary artery disease in patients with chronic renal dysfunction [14].

Researchers have long debated the extent to which homocysteine should be considered as a risk factor for cardiovascular diseases, since according to some, only 50% of CVD can be explained by “classical” risk factors, and they say that “new” risk factors could significantly boost the CVD predictive power [2]. But this has been widely criticized and there are other authors who show that up to three quarters of coronary heart disease (CHD) events, if not more, could be attributed to “classical” risk factors [2]. For the purpose of use as a screening tool, a risk factor should be strongly and causally associated with the target disease, and many authors doubt whether such a relationship between homocysteine and CVD exists [2].

The Framingham risk score (FRS), known as an important instrument in predicting coronary artery disease in patients with traditional risk factors, such as dyslipidaemia, hypertension, diabetes mellitus (DM), and smoking, seems to have underestimated the coronary artery disease risk in individuals with high homocysteine plasmatic levels [15]. Research has indicated towards a relationship between moderately elevated homocysteine levels and the risk of CVD (coronary, heart, cerebrovascular and peripheral artery diseases) [2]. The homozygous mutation of C‚S can cause severe hyperhomocysteinemia where homocysteine concentration is up to 40-fold of the normal levels. This disease occurs in approximately 1 of 100,000 live births [2]. When untreated, a vascular event (stroke, myocardial infarction, other thromboembolic complication) occurs in about half of these patients before the age of 30 [2]. Another cause of rare, genetically mediated severe hyperhomocysteinemia is due to homozygous mutations of MTHFR. People with these mutations have been noted to have premature cardiovascular diseases [2]. But a large meta-analysis showed the lack of statistically significant association between MTHFR mutations and coronary heart disease except in Middle East and Japan, where it portrayed statistical significance [2].

Homocysteine is known as an independent risk factor for atherosclerosis [16]. Arteriosclerosis is defined as a continuous inflammatory damage to the arterial intima with increased permeability to plasma, deposition of plasma lipids in plaques and fibrosis and calcification of plaques [15]. The correlation between hyperhomocysteinemia and atherosclerotic disease was first proposed more than 40 years ago. It was first identified by McCully in 1969. Atherosclerosis is the most common pathological process that leads to cardiovascular diseases such as myocardial infarction (MI), heart failure, stroke and claudication [13]. Several cross-sectional and case control studies have pointed towards a clear correlation between total serum homocysteine and the incidence of coronary, carotid, and peripheral vascular disease [17]. On the contrary, a systemic review of 12 randomized controlled trials on 47,429 subjects was carried out to discover the effectiveness of homocysteine lowering interventions. Unfortunately, homocysteine lowering interventions did not show any significant effect on myocardial infarction, stroke or death by any cause when compared to a placebo [17]. Homocysteine can mediate the formation of cardiovascular disease by several different mechanisms such as its adverse effects on vascular endothelium and smooth muscle cells with resultant alterations in subclinical arterial structure and function [18]. Some of the presumed mechanisms of these effects include an increase in proliferation of vascular smooth muscle cells, endothelial dysfunction, oxidative damage, an increase is synthesis of collagen and deterioration of arterial wall elastic material [18]. Examination of the effect of homocysteine on CRP expression and investigation on the related mechanism in vascular smooth muscle cells (VSMCs) revealed that homocysteine significantly induced mRNA and protein expressions of CRP in VSMCs both in vitro and in vivo [16]. Homocysteine augmented NR1 subunit (of N-methyl-D-aspartate receptor (NMDAr)) expression, while MK-801 reduced homocysteine induced CRP expression in VSMCs. The study demonstrated that homocysteine is capable of initiating an inflammatory response in vascular smooth muscle cells by stimulating CRP production, which is mediated through NMDAr-ROS-ERK1/2/p38-NF-κB signal pathway. These findings provided new evidence for a role of homocysteine in pathogenesis of atherosclerosis [16].

Using 70 participants (70 patients undergoing coronary angiography at Kasturba Hospital, Manipal University) Shenov et al. [10] showed that homocysteine is implicated as an early atherosclerotic promoter. Fasting serum homocysteine levels in CAD (Coronary artery disease) patients were significantly higher than patients without coronary artery disease (p < 0.001) [10]. Also homocysteine levels correlated significantly with increasing severity of coronary artery disease (p < 0.001). According to this paper, the most common and plausible mechanism for increased risk of CAD are endothelial dysfunction thought to occur primarily from changes in vascular endothelial compliance and platelet coagulation changes that promote cardiovascular disease [10]. In various in vitro studies, homocysteine was proved to trigger proliferation of vascular smooth muscle cells. It also has role in increasing the activity of HMG Co A reductase which in turn increases cholesterol synthesis [10]. An increased cholesterol level promotes atherosclerosis and hence it is a risk factor for CAD. Serum levels of homocysteine were found to be significantly higher in CAD than in non CAD subjects. Increased serum homocysteine levels positively correlated with severity of CAD [10]. But the authors assert too that there is a correlation between homocysteine and coronary artery disease, despite the fact that every research, including this one, has its limitations. Carotid intima-media thickness (IMT) is a well-accepted non-invasive marker of subclinical atherosclerosis [19]. The role of homocysteine in endothelial dysfunction is thought to be mediated by mechanisms including oxidative stress, nuclear factor-kb (NF-kb) activation, inflammation, and inhibition of endothelial nitric oxide synthase (eNOS) [19]. While several observational studies have reported weak positive associations between total homocysteine concentration and carotid IMT in the non-diabetic population, few cross-sectional studies address this association in the context of diabetes mellitus [19]. The following study observed the correlation in the case of diabetic patients. Although the data failed to include a control group without type 1 diabetes, in 599 Type 1 diabetic patients from DCCT/EDIC cohort, plasma total homocysteine levels were similar to those established for the general population, and correlated with numerous demographic and clinical parameters [19]. In multivariate analyses, significant correlations were maintained for age, diastolic blood pressure, and renal function. Plasma total homocysteine levels also correlated with common and internal carotid IMT measurements obtained approximately one and seven years later, but did not correlate with IMT progression as defined by the difference between these two determinations [19].

Investigators have reported a significant association of serum homocysteine concentration with different indices of arterial stiffness such as pulse pressure and aortic stiffness as assessed by carotid-femoral Pulse Wave Velocity (PWV) in the general population [18]. The carotid-femoral PWV was found to be significantly higher in the high homocysteine group than in the normal homocysteine group (*P* = 0.01), however there was no difference in carotid-radial PWV between the high homocysteine group and the normal homocysteine group [18]. Linear regression analysis revealed that homocysteine levels were significantly related to carotid- femoral PWV (*P* < 0.001) whereas no association was found with carotid-radial PWV [18].

The possible mechanisms explaining the relationship between hyperhomocysteinemia and aortic stiffness are not yet fully well established. Main hypotheses based on this investigation are that homocysteine plays a potential role in remodelling of the arterial wall leading to vascular damage [18]. This study as well as the one preceding it also stated that elevated homocysteine levels may have enhanced oxidative stress and inflammation of vascular endothelial cells and reduced the production and bioavailability of nitric oxide (a strong relaxing factor) by the endothelium [18]. There is also a strong evidence that oxidation is part of the mechanism attributed to increased homocysteine and atherosclerosis [10]. Thus we see a common belief across many papers that an inflammatory response could be in play.

In an experimental study on mini pigs, mild hyperhomocysteinemia was found to cause an arterial, site-dependent deterioration of the elastic structure involving metalloproteinase- related elastolysis [18].

Hyperhomocysteinemia has also been shown to be associated with a higher risk of venous thrombosis [2]. Increased homocysteine level has shown a predilection towards promotion of platelet adhesion to endothelial cells and has also been associated with higher levels of prothrombotic factors for example, β-thromboglobulin, tissue plasminogen activator and factor VIIc [18]. These lead to the augmentation of thrombus formation. In addition, it is possible that enhanced arterial stiffness in hyperhomocysteinemia might be attributed to homocysteine related LDL atherogenesis, like small particle size of LDL and its oxidative modification [18]. According to a research by Xie et al. [20] where RBCs from healthy adults were treated with Homocysteine (8, 20, 80, 200, 800 μmol/L) for 24 hours, homocysteine treatment dose dependently enhanced phosphatidylserine exposure and consequently the pro-coagulant activity of RBCs. Homocysteine also elevated the formation of pro-coagulant red blood cell-derived micro-particles, with statistical significance at 800 μmol/L of homocysteine [20]. In vitro studies indicate that homocysteine may have a harmful effect on endothelial cells, increasing coagulation, and proliferation of smooth muscle cells. However, homocysteine doses given in many in vitro studies far exceed pathological homocysteine levels in humans [2]. This has to be duly noted in all the future research carried out in this field and proper adjustment is a dire necessity to get appropriate and comparable results.

A separate study [17] involving the analysis of men aged 65 years or older, carotid RI (Resistive Index) has shown a significant degree of association with homocysteine. The data utilised carotid RI as a surrogate marker of cerebral peripheral artery resistance and pointed out a significant association between the index and homocysteine levels in elderly male patients with essential hypertension [17]. This indicates that increased serum homocysteine may be a marker of an increase in RI particularly in elderly patients with a greater risk of stroke [17]. Despite these evidences the fact that the subjects of this research were aged 65 and older, should be taken under consideration during speculation in terms of age related factor.

If we add both the genetic as well as nutritional factors, we may have another contributing factor at hand. Epigenetic directive of cardiovascular development and cardiovascular stem cell biology may be related to the cardiovascular disease predilection [5]. Nutrition and environmental exposures in utero or during periods of famine or any such critical periods in life, can cause epigenetic alterations in the expression of genes that contribute to disease risk of atherosclerosis, hypertension etc. later in life [5]. This outcome to some extent may be a result of dietary deficiency of folate, vitamin B12 or choline (a betaine precursor necessary for folate-independent methylation of homocysteine) since these are essential for methylation reactions that may epigenetically direct gene expression [5]. But in light of this, we do need to realize that folate supplementation is a common practice at present for pregnant women especially in developed countries, whereas cardiovascular diseases are more common in the developed world as opposed to the developing world.

Although it may be of lesser significance, we cannot completely overshadow this factor. Apart from being part of the antioxidant defence system, some vitamins also play a role as enzyme cofactors [13]. Vitamin B_6_, B_12_ and folic acid are essential cofactors in homocysteine-methionine metabolism. Therefore low vitamin B availability (B_6_, B_12_ and folic acid) leads to impaired re-methylation of homocysteine to methionine and thus to homocysteine accumulation [13]. Increased homocysteine levels were found to be associated with arteriosclerotic outcomes and risk of stroke in elderly individuals, and are considered as an independent risk marker for cardiovascular diseases [13]. However, lowering homocysteine levels by B-vitamin supplementation failed to demonstrate beneficial effects in cardiovascular diseases and this has been proven to be true in many other research works [13]. In addition, B vitamins were shown to reduce homocysteine without improving endothelial dysfunction or hypercoagulability [2]. Recent data also seem to indicate that homocysteine accumulates secondary to heightened oxidative stress associated with immune activation [13]. The association between cardiovascular diseases and homocysteine may result from deficiency of B vitamins or it may only alter vascular reactivity when folate is simultaneously low [2]. On the contrary, folate is associated with alteration in vascular reactivity without homocysteine concentration changes [2].

It is a universal truth that high blood pressure or hypertension leads to cardiovascular diseases. There are numerous factors contributing towards the development of hypertension, but the association of homocysteine with blood pressure deserves attention because blood pressure may mediate part of the cardio toxic effect of homocysteine [21]. A causal link exists between homocysteine and blood pressure and it is reinforced by experimental and animal studies that have reported a rise in blood pressure as a consequence of induced hyperhomocysteinemia [21]. Homocysteine may elevate blood pressure through numerous mechanisms such as its effect on vascular endothelial integrity [21]. Homocysteine administration has shown to cause direct endothelial cell injury in vitro and in animals, as stated before. Homocysteine induced oxidative stress to endothelium and reduced available nitric oxide (a potent vasodilator) in cell culture studies [21]. Observations in humans showed impairment of endothelium-dependent vasodilation in temporary or chronic hyperhomocysteinemia [21].

Homocysteine has been positively associated with both diastolic and systolic blood pressure. In case of homocysteine concentration increase of 5 μmol/L (about 1 SD), diastolic and systolic blood pressure in men increased by 0.5 and 0.7 mmHg, respectively [21]. In case of women, the correlation of homocysteine and blood pressure was stronger, with 0.7 and 1.2 mmHg increase in diastolic and systolic blood pressure, respectively [21].

To allow for nonlinearity, homocysteine was categorized into quintiles: The trend in the risk of hypertension with increasing homocysteine quintiles was significant only in women (p for trend = 0.0001) [21]. The homocysteine-cardiovascular disease association was slightly strengthened in women, but when the highest and the lowest quintiles of homocysteine were compared, risk of hypertension showed a threefold increase and a twofold increase in women and men respectively [21]. The correlation of homocysteine with prevalent cardiovascular disease has been examined with and without adjusting for blood pressure. Upon omission of blood pressure, the association was slightly strengthened in women, but there was little or no change in case of men [21].

An article originally published in Polish on Endothelial dysfunction in patients with primary hypertension and hyperhomocysteinemia had some important content. It stated the wide acceptance of the fact that endothelial dysfunction happens to be the basis of the development of cardiovascular diseases, including hypertension [22]. Endothelial dysfunction in the form of impaired vascular expansion is the major concern with regard to hypertension [22]. Along with the effects of hyperhomocysteinemia mentioned before, this study indicates that it adversely affects the biosynthesis and function of vasodilator factors in the vascular wall, which in turn contributes to endothelial cell division inhibition with intense myocyte proliferation and migration, and impairment of production of extracellular matrix components [22]. As mentioned earlier, high levels of homocysteine and its derivatives add to the process of modification of LDL and HDL particles, inflammation, coagulation disorders as well as fibrinolysis [22]. Hyperhomocysteinemia may lead to biochemical effects on endothelium and cause damage to endothelial cells, diastolic dysfunction of vessels and reduction of flexibility due to its influence on vascular wall remodelling [22]. These mechanisms may lead to an increase in blood pressure and strengthen the development of hypertension and damage body organs in patients with this disease [22].

The question therefore exists if homocysteine is a biomarker or a risk factor? Current guidelines have not classified homocysteine as cardiovascular disease risk stratification. The analyses by Veeranna et al. [14] prospectively validated and showed the incremental value of homocysteine level in predicting adverse cardiovascular disease events beyond the FRS. Therefore this paper states that homocysteine fulfils the criteria to classify it as a “novel” marker [14]. Although lowering homocysteine levels in individuals with pre-existing cardiovascular disease has not shown any benefit, medications as part of a primary prevention strategy need to be evaluated further for confirmation [14]. Therefore, it seems unfair to underestimate the utility of homocysteine in cardiovascular disease risk prediction solely because interventions to lower plasma homocysteine levels have not shown a favourable outcome regarding the risk of cardiovascular disease incidence [14]. Yet there is always room for more research to validate homocysteine as a risk factor and this is absolutely necessary for the sake of solid evidence.

On the other hand, such issue might be alarming. Some recent studies suggest that homocysteine levels may increase secondary to the occurrence of a cardiovascular disease and/or due to the presence of atherosclerosis [2]. Subjects with reduced renal function showed elevated homocysteine concentrations, which suggested that vascular disease may impair renal function, in turn leading to hyperhomocysteinemia [2]. But other findings showed that hyperhomocysteinemia is a predictor of cardiovascular disease in patients with renal failure as well as chronic stable renal transplant recipients independently of renal function and this is contradictory to the assumption that hyperhomocysteinemia is caused by renal dysfunction [2].

Even though it is possible that the abundance of published studies that show a positive correlation may reflect publication bias it is also likely that the negative studies are false negatives due to a lack of methodological or statistical power or random error [4]. A systematic review of studies with the same types of patients and controls and the same methods and outcome events may contribute towards a more accurate estimate of the association between homocysteine and vascular risk [4]. Furthermore, as discussed previously, the numerous positive results of retrospective studies may have been a result of consistent bias since homocysteine levels were usually measured after the acute vascular event and that could be the reason behind higher levels of homocysteine [4]. This is quite possible, since it has been noted to be an issue in most papers and has been speculated in many cases.

In an effort to see a cause and effect relationship, we carried out experiments in control and 10 weeks spontaneously hypertensive (SHR) rats. The rats were anesthetized and a microdialysis probe was inserted in paraventricular nucleus. The fluid was then aspirated for catecholamine estimation. Figure 2 shows that catecholamine concentration was higher in SHR rats. Once the homocysteine was infused through this probe, the level was significantly higher in SHR rats as compared to control animals (Figure 3). The SHR animals showed depressed cardiac contractility. The Table 1 shows the ventricular dP/dt in control and stroke prone SHR rats; the values are significantly depressed in experimental rats. Our results are consistent with a view that homocysteine through the release of catecholamines can produce detrimental effect in brain and cardiovascular system.

**Figure 2:** **Norepinephrine concentration (nmol/L) in paraventricular nucleus.** Mean value of 6 experiments (*p value < 0.05).

**Figure 3:** **Norepinephrine concentration (nmol/L) in paraventricular nucleus following homocysteine (20 μM) infusion.** The values are mean of 6 experiments. *p < 0.05.

**Table 1:** **Effect of homocysteine (20 μM) infusion on cardiac contractility**

Cardiac contractility dP/dt (mmHg/sec)	
Control	SHR
1622 ± 120	1056 ± 182*

Results are means ± SE of 6 experiments. Homocysteine was infused through microdialysis probe in paraventricular nucleus and then cardiac contractility was measured through a Miller catheter.

*P < 0.05.

## Conclusion

The published literature indicates that homocysteine is an independent cardiovascular disease risk factor modifiable by nutrition and exercise. However, it is now widely accepted that food sources alone cannot consistently supply the levels of nutrients necessary to sustain optimal homocysteine metabolism. In fact, emerging studies are uncovering novel nutritional strategies for lowering high homocysteine levels offering new possibilities for preventing cardiovascular disease.

The speculation of this peculiar correlation continues to contribute to the perplexity of the scientific society. Though most research work suggests a relationship, yet there seems to be other evidence that still prevents its inclusion as a biomarker. With every ten steps forward, we might have to face a step or two backward, but this should only further increase the enthusiasm of research in this field. This field definitely needs more research input until a definitive proof is available to cast off any shadow of doubt regarding the correlation between homocysteine and cardiovascular disease. Nevertheless, the present review should provide some insight into the role of homocysteine in the development of cardiovascular disease summarizing both central and peripheral effects of homocysteine. The authors feel that it is necessary to combat the ill effects of hyperhomocysteinemia as it has a pivotal influence on the pathology of the diseased process.
